# Performance Art Video Action Management Oriented to 6G Wireless Transmission Technology

This article has been retracted.

**DOI:** 10.1155/2022/1649455

**Published:** 2022-10-07

**Authors:** Yong Wang, Nam-gyu Cho

**Affiliations:** Department of Performance Art Management, Sangmyung University, Seoul 03015, Republic of Korea

## Abstract

With the development of 5G communication networks, the development prospects, capability requirements, and key technologies of the next-generation communication system 6G have become new hotspots. This article expands the coverage of the communication system through 6G, realizes the wireless transmission technology, builds the ideal of an intelligent mobile society everywhere, and analyzes the development trend of 6G technology, the challenges it faces, and the possible wireless transmission technology. Wireless transmission technology is widely used in various fields of production and life. Its various technical requirements and terminal energy limitations restrict the application and development of communications. This article focuses on the high-efficiency optimization scheme that combines 6G wireless transmission technology to improve the utilization efficiency of network resources. In addition, this thesis also discusses video action management in public performance art. Based on public performance art, the research on video action recognition can be summarized into three levels from simple to complex according to the content of the action, namely mobile vision, action vision, and action vision. Video action vision is currently being studied. In the recognition process, most of the action frame information in the video is repetitive or has a low correlation with action recognition, which not only increases the complexity of calculation but also affects the accuracy of action recognition. In the process of feature selection and understanding, the main methods include characterization fusion and research based on gesture features. Based on the introduction of 6G wireless transmission technology, this article introduces the technological development of 6G network, which promotes the rapid development of public performance art video action management.

## 1. Introduction

The 5G communication system has been commercialized, and its development has been deeply integrated with the real economy to form a good 5G industrial ecology. In this context, international organizations and governments plan to carry out research on 6G communication systems [1]. Currently, 6G does not have a unified definition, but there are several preliminary consensuses on application scenarios, technical trends, and key indicators [2]. We sorted out the overall vision of 6G, 8 business application scenarios, and corresponding indicator requirements and put forward some important technical indicators of 6G [3]. Wireless transmission technology is the main technical way to achieve the main indicators of 6G [4]. The problems of the wireless transmission technology used in the existing 5G are still significant, and the wireless transmission technology needs to be further improved [5]. This paper studies energy efficiency optimization under wireless transmission technology scenarios, focusing on MTC energy consumption and wireless transmission technology, analyzes related typical processing methods, and proposes improved and innovative solutions based on future work [6]. In order to further solve the efficiency problem of MTC, this article will introduce the data integration strategy based on wireless transmission technology [7]. In addition, for energy consumption models with different delay requirements, this paper proposes a power selection scheme based on the maximum efficiency target and conducts efficiency optimization research in this scheme [8]. This article applies wireless transmission technology to video operation management in public performance art. The development process of video action recognition can be summarized as mobile vision, action vision, and behavior vision [9]. So far, video actions are still in the stage of action vision research, that is, by extracting some features from training data, using supervised or unsupervised training to create classification models, extracting features from new data, and sending them to the model to obtain classification results [10]. From the perspective of video action recognition input under public performance art, video action recognition under the framework of public performance art has developed from action recognition in images to human action recognition in the video process [11]. Recognition is the process of learning and understanding human behavior by processing and analyzing the original images or sequences collected by sensors. Generally speaking, the detection technology based on feature extraction is a technology with better comprehensive performance [12]. We obtain the human motion model, establish the projection relationship between the video content and the motion type description, and realize the computer understanding of the video [13–16].

On the whole, video action recognition has evolved from simple hand or foot action interaction to the analysis and acquisition of human body movements. Among the subtle differences, the recognition rate of subtle movements such as facial expression recognition and gesture recognition will become higher and higher. Through the development of 6G communication system and wireless transmission technology, the analysis of video behavior in public performance art will lay the foundation for the development of public performance art in the future.

## 2. Related Work

The literature proposes that with the continuous emergence of new multimedia services and the current research status in China, new challenges are presented to the design of future 6G mobile networks [17]. Aiming at the business optimization problem in wireless transmission technology, an efficient and low-cost optimization algorithm is proposed and solved through a design algorithm [18]. The simulation results show that the cooperative multimode transmission strategy is feasible [19]. The literature proposes the relationship between video service management and wireless transmission technology and introduces the advantages of video service management and wireless transmission technology in terms of network delay, efficiency, and power consumption [20]. The literature puts forward the application of broadband wireless transmission technology in low and high frequency and discusses the research direction of broadband wireless transmission technology in the future [21]. The literature introduces a recognition method that uses a computer to process and analyze the original image or sequence image data collected by the sensor so that the computer can understand the video [22]. The literature proposes that the form and content of the action are complementary to each other, and video movement management provides a more comprehensive strategy and method for the overall performance art arrangement innovation, and it provides a theoretical reference for further research [23–26].

## 3. Research on Wireless Transmission Technology for 6G Multimedia Services

### 3.1. The Overall Frame Structure of the Wireless Transmission Network

#### 3.1.1. 6G Wireless Backhaul Network Distributed Architecture

The macro base station is located in the center of the macro cell with a radius of *R* and controls the infinite backhaul of the small cell base station within the coverage of the macro cell [27–30]. Due to the strong directionality of millimeter waves, the interference of adjacent nodes can be ignored. In order to realize the transmission of wireless backhaul services in 5G ultradense cellular networks, a distributed wireless backhaul network architecture is usually used.

Since millimeter wave has large path loss and obvious dispersion effect, it is assumed that the hop distance of wireless transmission does not exceed *D*0, that is, each small cell base station can only connect to the small cell base station with the base station as the center of the circle and *D*0 as the radius. . Because the future 5G cellular network will be dense, even ultracompact, by correctly locating the backhaul gateway, we can assume that the normal base station of *N* small cells can send data to the corresponding backhaul gateway node.

#### 3.1.2. Software-Defined Network Architecture

At present, the definition of software grid technology has already had a certain basic research [31–34]. The SDN network architecture combining “backbone + access network” and satellite-borne optoelectronic hybrid switching is shown in Figure 1.

Through the control plane sending rules, the various modules of the plane data network can be programmed by collecting topology information and status feedback of the plane data network nodes. The controller serves as the data plane management module, including the use of photoelectric hybrid switches to adapt to changes in the network scene. Here, the data plane management module is mainly responsible for the configuration of the satellite orbit height.

### 3.2. Heuristic Energy Efficiency Optimization Algorithm for Different Time Delay Scenarios

#### 3.2.1. Energy Consumption Model

Since the power consumption of the MTC terminal is mainly in data transmission, this article considers the power consumption of the MTC terminal in data transmission [35–37]. Therefore, when the terminal transmits bit data and transmits power, the following power consumption formula is used to evaluate the power consumption:

(1) $$\begin{array}{c} E_{T}\left(l,p\right)=p\times \frac{l}{B\times \log_{2}\;\left(1+SNR\right)}\text{.} \end{array}$$

Among them, *l* represents the data packet size, *p* represents the terminal transmission power, *B* represents the wireless resource transmission bandwidth, and SNR represents the signal-to-noise ratio at the receiver.

The specific calculation formula is as follows:

(2) $$\begin{array}{c} SNR=\frac{p\times h_{d}^{2}}{N_{0}B}\text{,}\\ \begin{array}{c} p\leq p_{\max\;,}\\ SNR\geq r_{0}. \end{array} \end{array}$$

*N*_0_ represents the noise power spectral density, *r*_0_ represents the received signal-to-noise ratio threshold, and *h*_*d*_^2^ represents the limit range of the communication distance of the MTC remote communication terminal.

Under the constraints of the maximum transmission power *p*_max_ and the signal-to-noise ratio *r*_0_, the expression for the communication range *d*_max_ of the MTC terminal is obtained as follows:

(3) $$\begin{array}{c} d_{\max}={\left(\frac{10^{-3.06}p_{\max}}{r_{0}N_{0}B}\right)}^{1/7.52}\text{.} \end{array}$$

In the current network environment, the MTC terminal is fixed and has no mobility. In this case, only other MTC terminals within the communication range *d*_max_ can directly communicate with it. The expression is as follows:

(4) $$\begin{array}{c} DCDS_{i}=\left\{MD_{r}\;|\;r=1,2,\ldots ,n_{i},且d_{ij}\leq d_{\max}\right\}\text{,}\\ D_{i}=\left\{dcd_{ir}\;|\;r=1,2,\ldots ,n_{i}\right\}\text{.} \end{array}$$

Among them, DCDS_*i*_ is MD_*i*_ which is the corresponding set of direct communication terminals, representing the Euclidean distance from MD_*j*_ to MD_*i*_, *n*_*i*_ is the total number of MTC terminals contained in DCDS_*i*_, and dcd_*ir*_ is the communication distance between MD_i_ and the rth MTC in DCDS_*i*_.

Therefore, under the current scenario energy consumption model, this article refers to the set of all possible transmission powers as the transmission power selection set, and its set expression is as follows:

(5) $$\begin{array}{c} TPS_{i}=\left\{p_{ir}\;|\;r=1,2,\ldots ,n_{i}\right\}\text{.} \end{array}$$

Among them, *p*_*ir*_ is MD_*i*_, which is the transmission power corresponding to the data sent to the *r*th terminal of its direct communication terminals set under the current energy consumption model based on the maximum energy efficiency target of one hop. Combining equation (1), the communication energy consumption CEC_*i*_ corresponding to MD_i_ when the transmission power is *p*_*ir*_ is as follows:

(6) $$\begin{array}{c} CEC_{i}=p_{ir}\times \frac{l}{B\times \log_{2}\;\left(1+q_{ir}\times p_{ir}\right)},p_{ir}\in TPS_{i},r\in \left\{1,2,\ldots ,n_{i}\right\}\text{.} \end{array}$$

Among them, *q*_*ir*_ is the ratio of channel gain squared to noise power, and its calculation formula is

(7) $$\begin{array}{c} q_{ir}=\frac{h_{d}^{2}\left(d_{c}d_{ir}\right)}{N_{0}B}\text{.} \end{array}$$

#### 3.2.2. The Problem of Wireless Resource Allocation

This article defines the concept of the equivalent rate *v*_*i*_ and proposes the ratio of the equivalent rate to MD_i_ delay in the sense of MD_*i*_ delay, which reflects the speed at which data reaches the sink node from MD_*i*_ at the beginning of network communication, and its specific calculation formula as follows:

(8) $$\begin{array}{c} v_{i}=\frac{l}{wt_{i}+ct_{i}}\text{.} \end{array}$$

Among them, *l* is the amount of data sent, wt_*i*_ is the waiting delay from the start of network communication to its data transmission and the transmission delay of data sent and relayed from other terminals to the receiver node. This article converts the transmission sequence of the terminal corresponding to the wireless resource allocation scheme into its numbered sequence vector, which is recorded as *A*, and the specific form is as follows:

(9) $$\begin{array}{c} A=\left(a_{1},a_{2},\ldots ,a_{i},\ldots ,a_{N}\right),a_{i}\in \varphi \text{.} \end{array}$$

Among them, *a*_*i*_ represents the terminal number corresponding to the MTC terminal, and its expression is as follows:

(10) $$\begin{array}{c} B=\left(b_{1},b_{2},\ldots ,b_{i},\ldots ,b_{N}\right),i\in \varphi \text{.} \end{array}$$

Among them, *b*_*i*_ indicates that the *i*-th MTC terminal in the number arrangement sequence vector *A* uses RB resources to transmit its own data. The expression of *b*_*i*_ is

(11) $$\begin{array}{c} b_{i}=\left(b_{i1},b_{i2},\ldots ,b_{ij},\ldots ,b_{ih_{i}}\right),h_{i}-1<H\text{.} \end{array}$$

In this article, the number of sink nodes is recorded as zero. For 1 < *j* < *h*_*i*_, *b*_*ij*_ in *b*_*i*_ indicates that the data of MD_*ai*_ is at the *j* − 1th hop, and the relay responsible by MD_*bij*_ is sent at the second hop. Therefore, the *b*_*ij*_ expression is

(12) $$\begin{array}{c} b_{ij}\left\{\begin{array}{c} =a_{i},j=1\text{,}\\ \in \left\{\left\{1,2,\ldots ,N\right\}-\left\{a_{i}\right\}\right\},1<j<h_{i}\text{,}\\ =0,j=h_{i}\text{.} \end{array}\right. \end{array}$$

From equations (10) and (11), combined with the rate formula (2), this paper gives the expression of the transmission delay ct_*ai*_ of MD_*ai*_ as follows:

(13) $$\begin{array}{c} ct_{a_{i}}=\overset{h_{i}-1}{\underset{j=1}{\sum }}\;\frac{l}{v\left(p_{b_{ij}},d_{b_{ij},b_{i\left(j+1\right)}}\right)},p_{b_{ij}}\in TPS_{b_{ij}},d_{b_{ij},b_{i\left(j+1\right)}}\in D\text{.} \end{array}$$

If the total number of RBs in the current network is *M*, the MTC terminal corresponding to the first *M* number in the numbering vector A has no waiting time delay in terms of delay composition. Therefore, the last MTC terminal among the corresponding MTC terminals has a waiting time delay. For the MTC terminal with waiting time delay, the *M* currently using RB resources is the minimum time delay of the terminal currently using resources. Therefore, for MD_*ai*_, the expression of its waiting time delay wt_*ai*_ is

(14) $$\begin{array}{c} wt_{a_{i}}=\left\{\begin{array}{c} 0,1\leq i\leq M\text{,}\\ \min_{a_{j}\in \left\{\forall i-M\leq j<i\right\}}\left(wt_{a_{j}}+ct_{a_{j}}\right),M<i\leq N\text{.} \end{array}\right. \end{array}$$

In the current network scenario, the delay calculation of the MTC station is measured by the corresponding delay index. This article uses the time index of each station multiplied by the corresponding equivalent rate data as the utility function. The function form is as follows:

(15) $$\begin{array}{c} v_{all}=\overset{N}{\underset{i=1}{\sum }}\;\left(\theta_{a_{i}}\times v_{a_{i}}\right)=\overset{N}{\underset{i=1}{\sum }}\;\left(\frac{\theta_{a_{i}}\times l}{wt_{a_{i}}+ct_{a_{i}}}\right)\text{.} \end{array}$$

Among them, *θ*_*ai*_ is the delay index corresponding to the *i*-th terminal in the number sequence vector that uses the resource to transmit its own data, and *v*_*ai*_ is the equivalent rate of the corresponding terminal. Combined with the definition of the equivalent rate, the corresponding equivalent rate is also required to be larger.

#### 3.2.3. Energy Consumption Issues

The above discussion is about wireless resource allocation in current network scenarios. Next, analyze the energy consumption in the current network scenario [38–41]. For MD_i_, the number of communications is unknown. For ease of expression, it can be recorded as cn_*i*_. Using the above energy consumption model and equation (5), this paper gives the expression of MD_*i*_ energy consumption EC_*i*_ as follows:

(16) $$\begin{array}{c} EC_{i}=\overset{cn_{i}}{\underset{g=1}{\sum }}\;\left(p_{ig}\times \frac{l}{v\left(p_{ig},d_{ig}\right)}\right),p_{ig}\in TPS_{i},d_{ig}\in D_{i}\text{.} \end{array}$$

Among them, TPS_*i*_ is the transmission power selection set, *D*_i_ is the direct communication distance set, *p*_*ig*_ and *d*_*ig*_ are the transmission power and corresponding communication distance during the *g*th communication, respectively. Therefore, the total energy consumption of all terminals of MTC is

(17) $$\begin{array}{c} E_{all}=\overset{N}{\underset{i=1}{\sum }}\;EC_{i}=\overset{N}{\underset{i=1}{\sum }}\;\left(\overset{cn_{i}}{\underset{g=1}{\sum }}\;\left(p_{ig}\times \frac{l}{v\left(p_{ig},d_{ig}\right)}\right)\right)\text{.} \end{array}$$

It can be seen from the above analysis that in the current scenario, the relay selection will affect the energy consumption and wireless resource allocation of the MTC terminal at the same time. Therefore, this article considers the two together, the smaller the energy consumption, the better, and the larger the weighted equivalent interest rate sum, the better. Therefore, this paper adopts the weighted equivalent rate and the ratio of *v*_all_ to the total energy consumption *E*_all_ as the final energy efficiency index. The overall energy efficiency expression is as follows:

(18) $$\begin{array}{c} EE_{all}=\frac{v_{all}}{E_{all}}\\ =\frac{\overset{N}{\underset{i=1}{\sum }}\;\left(\theta_{a_{i}}\times v_{a_{i}}\right)}{\overset{N}{\underset{i=1}{\sum }}\;EC_{i}}. \end{array}$$

It can be seen from this formula that the smaller the total energy consumption, the higher the corresponding weighted equivalent rate, and the higher the total energy efficiency of the network. Therefore, the maximum energy efficiency index can be used to deal with the energy consumption of the network. It is related to the wireless power consumption and resource allocation in the current scenario. In summary, the final energy efficiency optimization problem in this article can be specifically expressed as

(19) $$\begin{array}{c} \max_{a_{i}\in A,b_{i}\in B}\;\frac{\sum_{i=1}^{N}\left(\theta_{a_{i}}\times l/wt_{a_{i}}+\sum_{j=1}^{h_{i}-1}\left(1/v\left(p_{b_{ij}},d_{b_{ij},b_{i\left(j+1\right)}}\right)\right)\right)}{\sum_{i=1}^{N}\left(\sum_{g=1}^{cn_{i}}\left(p_{ig}\times 1/v\left(p_{ig},d_{ig}\right)\right)\right)}\text{.} \end{array}$$

The constraint condition of this optimization problem is that the number of MTC terminals in equation (8) is arranged according to the sequence vector in equation (16) and the corresponding communication path vector, and the transmission power corresponds to the transmission data. In the denominator, one group is selected from the corresponding transmission power equation (4), and the number of relays is determined by multihop communication in actual communication.

#### 3.2.4. Heuristic Optimization Scheme

In the above efficiency optimization problem, for any one of the MTC terminals, different transmission destination nodes choose to determine different transmission powers [40–42]. The set expression of *D*_toSN_ and *E*_res_ is

(20) $$\begin{array}{c} D_{toSN}=\left\{d_{i}\;|\;d_{i}=d\left(SN,MD_{i}\right),i\in \varphi \right\}\text{,}\\ E_{res}=\left\{E_{i}\;|\;i\in \varphi \right\}\text{.} \end{array}$$

Among them, the Euclidean distance from the aggregation node SN represents the current remaining energy.

If you want to register the currently selected relay node, relay must meet the following conditions:

(21) $$\begin{array}{c} \left\{{relay}_{i}{=relay}_{i}\in DCDS_{i}⟶\min_{r=1,2,\ldots ,n_{i}}\left(\frac{E_{ave\;}}{E_{r}}+d_{r}\right)\right\}\text{.} \end{array}$$

Among them, the corresponding group of direct communication terminals is the residual current power of the *i*-th terminal, and the calculation formula is as follows:

(22) $$\begin{array}{c} E_{ave}=\frac{\overset{N}{\underset{i=1}{\sum }}\;E_{i}}{N}. \end{array}$$

Among them, *E*_*i*_ is the current remaining energy of the *i*-th MTC terminal among all current MTC terminals.

### 3.3. Simulation Experiment Results and Performance Analysis

Based on the system delay model proposed under the multimodal transmission strategy, the influence of system parameters on the delay is compared through numerical simulation analysis. Under different popular deviations, the relationship between the delay of the optical fiber link and the AR/VR video content of the edge data center is consistent.

Due to the increase in storage capacity, more data needs to be sent to each data center. When the size of the small cell base station cache segment changes, for the edge data center, more data needs to be transmitted so as to avoid the increase of backhaul delay caused by playing video.

The power density of edge data centers increases with the increase of edge data center density. In the case of constant edge data center density, as the edge data center density increases, the greater the edge data center density, the greater the power consumption.

## 4. Realization of the Performance Art Video Action Management System under Computer Technology

### 4.1. The Overall Structure of the Video Action Management System Database

There are many main entities in the database, such as playing and recording alarm information, control information, users, management, and types. After analyzing the flow chart of the ER system, the next step is mainly to store information for each database entity.

The user information table is responsible for the content of user information related to the operation of the video information management system. The detailed table is shown in Table 1:

From Table 1, we can see the field name, field type, whether it is empty or restricted, and other related information.

The video information table is mainly responsible for the content management of video information. The detailed table is shown in Table 2:

From the video information table in Table 2, we can see the field name, field type, whether it is blank, and the corresponding data constraint information.

The video type table is responsible for content information related to the video type in the video information management system. The detailed table is shown in Table 3:

From the video type table in Table 3, we can see the field name, field type, whether it is blank or restricted, and so on.

The user play record table is mainly responsible for the video operation information of the video content management system. The detailed table is shown in Table 4:

From the user playback record table in Table 4, we can see that the corresponding data information includes the field name, field type, whether it is empty, and restricted conditions.

### 4.2. Recognition and Analysis of Performance Art Video Action Sequence

The experiment uses a certain song and dance action in a motion capture device as the data set and selects the combination of the 11th group of dance action steps as the sample data. By manually dividing and removing the initial preparation action and the final end action, 4 combinations of similar actions were confirmed.

As can be seen from Table 5, the first segmentation position is located in the 105th frame. During the preparation of the sequence of action frames, no action information will be lost. The movements between frames 105 and 218 are obvious. Under normal circumstances, they are mistaken for simple movements. Usually, small staggers and raising of the hind legs belong to a sequence of dance movements.

The difference between other automatic segmentation positions and unrelated actions or manual segmentation is small, so the correct segmentation result will be obtained. Since there are many misdivision positions in the initial division position, the difference limit between frame sequences and the difference limit between adjacent minimum and maximum values are added.

The comparison of the segmentation position after adding the constraint conditions is shown in Table 6.

The video frame sequence segmentation algorithm is mainly composed of the PCA algorithm and the clustering algorithm. Compared with other algorithms, the algorithm in this paper requires two measurement parameters, which can be divided into the precision rate and the recall rate.

The segmentation effect of the algorithm in this paper is compared with other algorithms, as shown in Table 7.

In the action sequence, *A*0 is a preparatory action and does not contain clear action information. In the table, we can see that the regular distance between *A*0 and other action sequences is very large, while the regular distance is relatively between other action sequences. Smaller, it is certain that similar actions will occur in other action sequences.

### 4.3. Strategic Analysis of Innovation in the Arrangement of Performance Art Works

#### 4.3.1. The Theme Style Center Is Prominent

In the performance of art works, it is important to choose what theme and how to run through the theme of the whole work. The style of the theme must be clear. When choosing the theme, we can choose hot issues. Contemporary society reflects social phenomena. Art comes from life. It can determine the theme of the work according to what people see, hear, feel, and perceive life. When determining the theme of the work, it determines the cultural connotation that the theme wants to convey. The works are passed on from generation to generation, which not only fully interprets the works but also has profound connotations, which are worthy of promotion, exploration, and learning.

#### 4.3.2. Characters Are Vividly Created

In general performance art works, characters are the main part of the work. Whether it is a work describing characters or things or the performer's own certain temperament and skills, it requires the choreographer and performer to deeply experience the character to be expressed so as to create a rich and vivid image in the work. For example, expressing emotions, characters and thoughts in stories, understanding and reflecting the inner spirit of the works, and highly mastering dance skills are characterized by complexity and strong expression.

#### 4.3.3. The Concentration of Special Features Is Obvious

Public performance art works have a strong particularity. The operation, difficulty, and transition of each special event have obvious style characteristics and technical skills. For example, rhythmic gymnastics is softer, and cheerleaders can show more momentum. Choreographers need to make full use of these characteristics to display their works and maximize the performers' own technical advantages.

#### 4.3.4. Musical Works Are Integrated

In the public performance art works of the Graduate School of Sports, music is not an accessory that occupies an important position in the choreography structure. It is an important part of the compilation of works. Music is a work that is felt from another organ (ear) of the human body. In the choice of music, make full use of the theme, thoughts, and feelings of the work, use music to describe the characters deeply, make the image of the dance emerge, shape the stage environment, express the dance scene, and make full use of the music to express the emotional communication between the characters. It must not only conform to the characteristics of the selection method of the work but also perfectly show a series of action content.

#### 4.3.5. The Stage Beauty Effect Is Wonderful and Dazzling

In public art works, the beauty of dance can help you organize the creativity of your work. The exquisite stage design can instantly attract the attention of the audience. As a material means, it allows people to intuitively feel the status of the work while allowing the audience to intuitively feel the context of the work while also giving the work more space. Therefore, choreography can render the atmosphere of the stage, set off the performance of the work, promote the development and completion of the plot of the work, and simulate and reproduce the image of specific objective things.

#### 4.3.6. Technology of Embellished Fashion

With the development of science and technology, modern science and technology have penetrated into various fields. In the field of dance, the form of the stage pays more and more attention to the integration of science and technology. This not only diversifies the form of expression of the work but also gives the work more space. Although science and technology are the products of modernization, when combined with history and the movements of classical characters, the audience can more fully enter the artistic conception and deepen the theme. For example, making full use of the combination of LED technology and the story of the work can provide a powerful means for the narrative of the story. The combination of light and shadow technology and work clothes can enrich dance performance. The combination of lighting technology and the content of the work creates a stage atmosphere of different atmospheres.

## 5. Conclusion

Wireless transmission is about to enter the 6G era. Large-scale wireless transmission technology, as one of its three application scenarios, has a very broad application prospect in production and life. For wireless transmission technology, communication requirements are different in different application fields. The problem of energy consumption optimization for high-efficiency services of wireless transmission technology is proposed. It uses two-step solution and related algorithms to solve the problem. The performance of the system model is analyzed through numerical simulation, and the solution and optimization problem of the multipath common transmission strategy is analyzed. As people's demand for wireless transmission technology increases, the professional action correction of video actions that are closely related to human life and the application of action recording under public performance art have promoted the development of video action recognition research from simple action recognition to complex video actions. The current goal is to identify the specific target in the video, and the next stage is to identify the purpose of the human body for certain types of actions. The application of static features cannot stably guarantee the positive effect of target recognition in various databases. Looking forward to the development of wireless transmission technology under 6G network technology, it can bring certain development to the video action management under the public performance art in the future.

## Figures and Tables

**Figure 1:** Architecture of 6G software defined network.

**Table 1:** User table.

Field name	Field type	Can it be empty	Restrictions
User _id	Int	Not null	Primary key constraint
User _name	Varchar (20)	Not null	Unconstrained
User _password	Varchar (20)	Not null	Unconstrained
User _register date	Date	Not null	Unconstrained
User _last login date	Date	Not null	Unconstrained
User _point	Bigint	Null	Unconstrained
User _account	Varchar (20)	Null	Unconstrained
User _e-mail	Varchar (30)	Not null	Unconstrained
User _state	Int	Null	Unconstrained
User _telephone	Varchar (11)	Null	Unconstrained
User _money	Float (8, 2)	Null	Unconstrained

**Table 2:** Video information table.

Field name	Field type	Can it be empty	Restrictions
Video _id	Int	Not null	Primary key constraint
Type _id	Int	Not null	Foreign key constraint
User _id	Int	Not null	Foreign key constraint
Video _title	Varchar2	Not null	Unconstrained
Video _desc	Varchar2	Null	Unconstrained
Video _point	Long	Not null	Unconstrained
Video _play count	Long	Null	Unconstrained
Video _upload time	Date	Null	Unconstrained
Video _last playtime	Date	Null	Unconstrained
Video _URL	String	Not null	Unconstrained
Video _size	Int	Not null	Unconstrained
Video _keywords	String	Null	Unconstrained
Video _check state	Int	Not null	Unconstrained
Video _money	Float	Null	Unconstrained

**Table 3:** Video type table.

Field name	Field type	Can it be empty	Restrictions
Type _id	Int	Not null	Primary key constraint
Type _name	String	Not null	Unconstrained
Type _create time	Date	Not null	Unconstrained
Type _update time	Date	Not null	Unconstrained
Type _desc	String	Null	Unconstrained
Type _creator	Varchar (100)	Not null	Unconstrained
Type _updater	Varchar (100)	Null	Unconstrained

**Table 4:** User play record table.

Field name	Field type	Can it be empty	Restrictions
Play_ id	Int	Not null	Primary key constraint
Video_ id	Int	Not null	Foreign key constraint
Use_ id	Int	Not null	Foreign key constraint
Play_ time	Date	Not null	Unconstrained

**Table 5:** Comparison of manual segmentation and automatic segmentation position.

Motion segment	Start frame	End frame	Auto segmentation result	Movement description
1	1	121	105	Preparatory action

2	122	291	218	Irrelevant movement of raising the leg after a small stagger
	292	351	357	

3	352	421	498	Irrelevant movement of raising the leg after a small stagger
	422	491		

4	492	555	621	Irrelevant movement of raising the leg after a small stagger
	556	607		

5	608	676	708	Raise your leg after a small stagger
	677	741	726	Irrelevant actions

**Table 6:** Comparison of segmentation positions with constraints added.

Motion segment	Start frame	End frame	Auto segmentation result	Movement description
1	1	121	105	Preparatory action

2	122	291	220	Irrelevant movement of raising the leg after a small stagger
	292	351	359	

3	352	421	500	Irrelevant movement of raising the leg after a small stagger
	422	491		

4	492	555	623	Irrelevant movement of raising the leg after a small stagger
	556	609		

5	610	678	726	Irrelevant movement of raising the leg after a small stagger
	679	741		

**Table 7:** Action sequence distance.

Action sequence	*A*0	*A*1	*A*2	*A*3	*A*4	*A*5
*A*0	0	320.7388	1903.5752	1610.4045	2586.0451	1197.0756
*A*1	562.2396	0	467.2324	363.5521	784.8847	233.9011
*A*2	3509.3267	534.9003	0	1 08.0586	50.6611	233.3638
*A*3	2773.5538	278.5315	70.5508	0	138.3108	233.3244
*A*4	4638.3942	898.7725	79.6685	219.3547	0	423.8952
*A*5	1878.3055	313.7522	108.2244	1 65.9044	170.7065	0

## Data Availability

The dataset can be accessed upon request.
